# The Application Effect of Jiawei Sanyu Shengjing Decoction Combined with High Ligation of the Spermatic Vein in Varicocele Male Infertility Patients

This article has been retracted.

**DOI:** 10.1155/2022/2629140

**Published:** 2022-08-18

**Authors:** Xiangpeng Lu, Hao Han, Zhi Biao Zhang, Hao Chen, Xingru Huang, Rui Zhang

**Affiliations:** ^1^The Second Affiliated Hospital of Heilongjiang University of Chinese Medicine, China; ^2^Heilongjiang Traditional Chinese Medicine Hospital, China

## Abstract

**Objective:**

To analyze the application effect of Jiawei Sanyu Shengjing decoction combined with high ligation of the internal spermatic vein in male infertility patients with varicocele (VC).

**Methods:**

106 male infertility patients with VC treated in our hospital from December 2018 to March 2019 were selected as examples. According to the length of stay, they were divided into the control group and observation group, with 53 cases in each group. High ligation of the internal spermatic vein was performed in both groups. On this basis, the observation group was treated with modified Sanyu Shengjing decoction, and the therapeutic effects of the two groups were compared.

**Results:**

The effective rate of 94.34% in the observation group was higher than 79.25% in the control group (*P* < 0.05). After treatment, the serum index level and sperm deformity rate in the observation group were lower than those in the control group, and the semen density and sperm activity were higher than those in the control group (*P* < 0.05).

**Conclusion:**

The treatment of VC male infertility with modified Sanyu Shengjing decoction combined with high ligation of the internal spermatic vein can effectively improve the number of sperm and reduce the density of semen.

## 1. Introduction

Varicocele is one of the common causes of male infertility, referring to the elongation and tortuosity of vine venous plexus in the spermatic cord [1–2]. The disease is more often seen in teenagers; according to the survey, the incidence of the disease is high, accounting for 10%~15% of normal men; clinical manifestations of scrotal swelling, local intermittent swelling pain, and other symptoms, if not timely treatment, may cause vague pain, dull pain, and another discomfort, leading to male testicular function decline, seriously affecting the daily life of patients [3–4]. Clinical drug treatment, such as flavonoids, and ockeyesin treatment can reduce clinical symptoms and improve sperm activity, but for patients with poor drug treatment effects, surgical treatment can be selected, which can restore the fertility of patients [5]. The high ligation of the internal spermatic vein used in this study achieved therapeutic results by cutting the venous blood reflux to the trailing vein [6]. In this study, 106 VC male infertility patients were admitted from December 2020 to March 2021 to explore the effectiveness of different treatment methods. The details are as follows.

## 2. Material and Methods

### 2.1. Clinical Data

A total of 106 male infertility patients with VC admitted to our hospital from December 2020 to March 2021 were randomly divided into the control group and observation group, with 53 cases in each group. The control group was at least 21 years old and at most 43 years old, and the mean age was 32.68 ± 1.15 years. The shortest duration is 1 year, and the longest is 10 years, on average 5.62 ± 1.05 years. Site of lesion is as follows: 21 left, 18 right, and 14 bilateral. The observation group was at least 22 years old and at most 45 years old, and the mean age was33.59 ± 1.68years. The shortest duration is 1 year, and the longest is 12 years, on average 6.08 ± 1.14 years. Lesion sites are as follows: 19 left, 25 right, and 9 bilateral. There was no significant difference between the 2 data groups (*P* > 0.05).

The following are the inclusion criteria: (1) can cooperate to complete semen and serum examination, (2) good compliance and no communication barriers, (3) sign the informed consent form, and (4) meet the varicocele criteria for male infertility [7].

The following are the exclusion criteria: (1) presence of serious diseases, (2) quit in the middle of the experiment, (3) azoospermatism, (4) blurring of consciousness, and (5) the vas deferens are impassable.

### 2.2. Method

In both groups, high ligation of the spermatic vein was taken. After anesthesia, supine position, head low foot height, CO_2_ pneumoperitoneum, maintenance pressure of 10~12 mmHg, 5 mm, 10 mm puncture holes on both sides of the rectus abdominis, and the cannula was placed. A T-shaped incision was made on the inner ring, the peritoneum was cut, the inner vein of the spinal cord was free, and double bandaged to observe whether there was a missing spinal cord. If there were bleeding points, the abdominal gas was discharged, the cannula was removed, and the wound was sutured after the operation. On this basis, the observation group added traditional Chinese medicine for treatment; the basic prescriptions were as follows: Fossilia Ossis Mastodi, *Salvia miltiorrhiza* Bunge 30 g each, *Schisandra chinensis* (Turcz.) Baill., *Lycium barbarum* L. 20 g each, Chuanxiong Rhizoma, *Paeoniae Radix* Rubra, Cornu Cervi Pantotrichum 8 g each, Foeniculi Fructus, *Bupleurum chinense* DC., *Carthamus tinctorius* L., *Amygdalus persica* L. 5 g, and 3 g *Commiphora myrrha* Engl. Soak in warm water for 30 min, 1 dose/d, take it in the morning and evening, and use it continuously for 3 months to observe the effect.

### 2.3. Observational Indicators

1. Treatment effect: after treatment, examination of semen showed that sperm morphology, quantity, and vitality are cured; the above index or standard changes, and the improvement is >50%; the above index or standard partially changes, and the improvement is 26% to 49% which is effective; no change compared with before treatment is invalid
2. Serum index: after 5 mL of venous blood was drawn in the morning and centrifugation, the serum levels of luteinizing hormone (LH), follicle-stimulating hormone (FSH), and androgen (T) were measured by the enzyme-linked immunosorbent method
3. Changes in semen therapy: the malformation rate, semen density, and sperm motility were analyzed by computer-assisted analysis

### 2.4. Statistical Analysis

It was analyzed by the SPSS 20.0 software. The, *n*/% is compared with the 2 tests. The *t*-test is indicated as m ± s. *P* < 0.05 shows a significant difference.

## 3. Result

### 3.1. The Treatment Effects of the Two Groups Were Compared

The effective rate of 94.34% in the observation group was higher than that of 79.25% in the control group (*P* < 0.05). See Table 1.

### 3.2. Comparing the Serum Indexes between the Two Groups

Before treatment, the comparison between groups (*P* > 0.05), and after treatment, the serum LH, FSH, and T levels in the observed group were lower than those in the control group (*P* < 0.05). See Table 2.

### 3.3. The Changes in Semen Treatment Were Compared between the Two Groups

Before treatment, for the comparison between groups (*P* > 0.05), the sperm malformation rate was lower than in the control group, and the semen density and sperm activity were higher than in the control group (*P* < 0.05). See Table 3.

## 4. Discussion

VC could cause oxidative stress factors and intratesticular environmental damage, hinder spermatogenesis, gather harmful substances at the testis, and reduce sperm quality, which is the main factor causing male infertility [8–9]. The results showed that the incidence of infertility in VC patients is >80%, and more clinical drugs and surgical treatment could effectively relieve clinical symptoms. Most operations use high ligation of the internal vein, and through the ligation of varicose cord vein, it blocks venous blood reflux and then relieves the pain phenomenon [10–11]. Studies have shown that although this operation can effectively improve the clinical symptoms and reduce the recurrence of testicular damage, some patients cannot recover the damaged testicular epididymis in a short time [12–13]. Therefore, accelerating the rapid recovery of testicular epididymal function is an urgent problem to be solved clinically [14].

In traditional Chinese medicine, VC belongs to the category of “Jin Shan” and “Jin Liu,” which is related to liver qi stagnation and meridian stasis. The treatment should be soothing the liver, not qi, and nourishing kidney replenishing essence is the main [15]. In this study, the male infertility patients with VC were treated with Jiawei Sanyu Shengjing decoction combined with high ligation of the spermatic vein. The results showed that 94.34% treatment response rate in the observation group was higher than 79.25% in the control group (*P* < 0.05). Posttreatment, the rate of sperm malformation in the observation group and the semen density and sperm activity were lower than that of the control group (*P* < 0.05). It is believed that this treatment regimen can effectively improve sperm morphology and improve sperm activity. Schisandra in traditional Chinese medicine belongs to NianFei SheChang medicine. It could promote the body's immune function, enhance the body's adaptability, and resist kidney disease. Lycium chinense is an invigorating Yin drug; it has the effect of enhancing immune function, antitumor, lowering blood lipid, and inhibiting the heart. The combination of the two has the effect of recuperation of blood qi, producing sperm and filling the pulp. Radix Paeoniae Rubra is a heat-clearing and blood-cooling (HCBC) medicine; it has the effect of antiarteriosclerosis, liver protection, and bacteria inhibition. Salvia miltiorrhiza has the effect of activating blood circulation, pure-minded, and treating boils. The combination of both has the effect of analgesia and dissipating blood stasis [16]. Rhizoma Chuanxiong is a medicine for promoting blood circulation and relieving pain. It has the effect of inhibiting the heart, expanding blood vessels, increasing coronary artery flow, and improving microcirculation. Foeniculum vulgare dulce belonged to Wenli medicine; it promotes gastrointestinal peristalsis, sex hormone-like effect. Bupleurum chinense belongs to Xinliang Jiebiao medicine; it has the effect of sedation, analgesia, alleviating liver injury, and promoting bile secretion. *Carthamus tinctorius* L. is a blood-activating medicine; it has the effect of reducing coronary resistance, improving peripheral microcirculation disorder, and relieving intestinal spasm. *Amygdalus persica* L. is a blood circulation and menstrual medicine; it can be anticoagulation, anti-inflammatory, analgesic, and antiallergic and can improve blood flow.*Commiphora myrrha* Engl. relieves pain and swelling; Os Draconis has the effect of calming, calm, and astringent. The combination of various drugs improves sperm activity and reduces the rate of sperm malformation. Serum index has some guiding significance for the prognosis of VC male infertility, in which serum LH can promote the conversion of cholesterol into sex hormone in gonadal cells. Serum FSH promotes follicle maturation. Serum T has androgen activity and has some protein assimilation. The results of this study showed that serum levels of LH, FSH, and T in the observation group were lower than those in the control group (*P* < 0.05). It is believed that this combination regimen can effectively improve the serum index of VC male infertility patients, which is similar to the results of the study by Lu and Chen [17].

## 5. Conclusion

In conclusion, for VC male infertility patients, high internal vein ligation combined with Jiawei Sanyu Sheng Jing decoction can effectively improve sperm quality and activity and can be promoted.

## Figures and Tables

**Table 1:** Comparison of treatment effects between the two patient groups (*n*, %).

Group	Number	Recovered	Obvious effect	Effective	Ineffective	Treatment effective rate
Observation group	53	21 (39.62)	15 (28.30)	14 (26.42)	3 (5.66)	50 (94.34)
Control group	53	18 (33.96)	13 (24.53)	11 (20.75)	11 (20.75)	42 (79.25)
*χ* ^2^						5.267
*P*						0.022

**Table 2:** Comparison of the serum indexes of the patients in the two groups ($\bar{x}\pm s$).

Group	Number	LH (IU/L)		FSH (IU/L)		T (nmol/L)	
		Before treatment	After treatment	Before treatment	After treatment	Before treatment	After treatment
Observation group	53	10.05 ± 1.54	4.69 ± 0.84^∗^	10.62 ± 1.84	6.05 ± 0.57^∗^	11.63 ± 2.51	14.62 ± 1.73^∗^
Control group	53	9.98 ± 1.18	5.88 ± 0.97^∗^	10.98 ± 1.89	7.91 ± 0.62^∗^	11.96 ± 2.64	16.94 ± 2.09^∗^
*t*		0.263	6.752	0.994	16.078	0.660	6.225
*P*		0.793	0.000	0.323	0.000	0.511	0.000

Note: compared with this group before treatment, ^∗^*P* < 0.05.

**Table 3:** Comparison of the changes in semen treatment between the two groups ($\bar{x}\pm s$).

Group	Number	The density of semen (×10^6^/mL)		Sperm activity (%)		Rate of treat sperm (%)	
		Before treatment	After treatment	Before treatment	After treatment	Before treatment	After treatment
Observation group	53	30.02 ± 1.54	50.62 ± 2.69^∗^	40.62 ± 5.91	55.18 ± 2.81^∗^	40.25 ± 6.59	31.02 ± 3.54^∗^
Control group	53	29.81 ± 1.47	45.18 ± 2.08^∗^	39.84 ± 5.82	50.24 ± 2.69^∗^	41.02 ± 6.91	34.69 ± 4.51^∗^
*t*		0.718	11.647	0.685	9.245	0.587	4.660
*P*		0.474	0.000	0.495	0.000	0.558	0.000

Note: compared with this group before treatment, ^∗^*P* < 0.05.

## Data Availability

The data used to support this study is available from the corresponding author upon request.
